# Enhancing microalga *Chlorella sorokiniana* CY-1 biomass and lipid production in palm oil mill effluent (POME) using novel-designed photobioreactor

**DOI:** 10.1080/21655979.2019.1704536

**Published:** 2019-12-28

**Authors:** Wai Yan Cheah, Pau Loke Show, Yee Jiun Yap, Hayyiratul Fatimah Mohd Zaid, Man Kee Lam, Jun Wei Lim, Yeek-Chia Ho, Yang Tao

**Affiliations:** a Department of Environmental Health, Faculty of Health Sciences, MAHSA University, Jenjarom, Malaysia; b Department of Chemical and Environmental Engineering, Faculty of Science and Engineering, University of Nottingham Malaysia, Semenyih, Malaysia; c Department of Applied Mathematics, Faculty of Science and Engineering, University of Nottingham Malaysia, Semenyih, Malaysia; d Fundamental and Applied Sciences Department, Centre of Innovative Nanostructures & Nanodevices (COINN), Institute of Autonomous System, Universiti Teknologi PETRONAS, Bandar Seri Iskandar, Malaysia; e Chemical Engineering Department, Universiti Teknologi PETRONAS, Seri Iskandar, Malaysia; f Centre for Biofuel and Biochemical Research, Institute of Self-Sustainable Building, Universiti Teknologi PETRONAS, Seri Iskandar, Malaysia; g Fundamental and Applied Sciences Department, Universiti Teknologi PETRONAS, Seri Iskandar, Malaysia; h Civil and Environmental Engineering Department, Universiti Teknologi PETRONAS, Seri Iskandar, Malaysia; i Centre for Urban Resource Sustainability, Institute of Self-Sustainable Building, Universiti Teknologi PETRONAS, Seri Iskandar, Malaysia; j College of Food Science and Technology, Nanjing Agricultural University, Nanjing, China

**Keywords:** Biofuel, Microalgae, Palm oil mill effluent, Photobioreactor, Wastewater

## Abstract

*Chlorella sorokiniana* CY-1 was cultivated using palm oil mill effluent (POME) in a novel-designed photobioreactor (NPBR) and glass-made vessel photobioreactor (PBR). The comparison was made on biomass and lipid productions, as well as its pollutants removal efficiencies. NPBR is transparent and is developed in thin flat panels with a high surface area per volume ratio. It is equipped with microbubbling and baffles retention, ensuring effective light and CO_2_ utilization. The triangular shape of this reactor at the bottom serves to ease microalgae cell harvesting by sedimentation. Both biomass and lipid yields attained in NPBR were 2.3–2.9 folds higher than cultivated in PBR. The pollutants removal efficiencies achieved were 93.7% of chemical oxygen demand, 98.6% of total nitrogen and 96.0% of total phosphorus. Mathematical model revealed that effective light received and initial mass contributes toward successful microalgae cultivation. Overall, the results revealed the potential of NPBR integration in *Chlorella sorokiniana* CY-1 cultivation, with an aim to achieve greater feasibility in microalgal-based biofuel real application and for environmental sustainability.

## 1. Introduction

Approximately 3–500 tonnes per year of microalgae biomass are required to produce microalgae consumer products in Asia-Pacific region [1]. Most of the cultivation plants are located in Asia like China, Taiwan and India [1]. Scientists from various countries are making tremendous efforts in developing efficient microalgae cultivation systems as microalgae are promising feedstocks for bioenergies and bioproducts productions. Effective microalgae cultivation requires a medium for nutrients and organics supply and adequate sunlight, CO_2_, temperature and aeration [2,3]. Comprehensive designs of cultivation system worked toward providing optimal growth conditions, eventually achieving high performance in biomass and lipid production. Open ponding system like circular and raceway ponds are conventionally applied for large-scale cultivations [4,5]. It offers a relatively good output of desirable yields at reasonable costs and could be incorporated in the industrial wastewater treatment if wastewater is used as a cultivation medium [6,7]. Yet, this culture is more susceptible to contamination risk, high evaporative loss and hindering sunlight penetration through the medium [8]. Closed photobioreactor could provide better regulation of the growth parameters, thus ensuring higher biomass yields than the open pond system [9]. Airlift, tubular, flat plate, bag, membrane and filtration-typed photobioreactors are well-recognized closed systems used for microalgae cultivation [10]. These photobioreactors work to promote the performance of microalgae biomass and lipid yields by enhancing optimal growth conditions. For instance, airlift photobioreactor promotes effective CO_2_ supply via bubbling in micron size, which encourages greater gas dissolution and mixing within the culture medium [11]. Tubular, flat plate and bag photobioreactors ensure maximal light received for boosting photosynthetic activity. Filtration photobioreactor works on attached growth cultivation system which is helpful for low cost and easy cell harvesting. Yet, there are pros and cons of these systems which requires further explorations. This is required to achieve effective microalgae cultivation for yields maximization, especially on a commercial scale. It is therefore important to incorporate an engineering approach into the microalgae cultivation system. In our previous studies, efforts have been focusing on the application of palm oil mill effluent (POME) as a cultivation medium for *Chlorella sorokiniana* CY-1 biomass and lipid production. Co-cultivation of *Chlorella sorokiniana* CY-1 and *pseudomonas* sp. had been studied as enhancement strategy. Carbon and nutrient supplementations were studied on a laboratory scale. Apart from changing the culture medium, the development of photobioreactor is also an important aspect to be explored as an enhancement strategy. Thus, in this study, we worked on enhancement of *Chlorella sorokiniana* CY-1 biomass and lipid production using novel photobioreactor (NPBR), with an aim to promote greater feasibility of microalgae cultivation and environmental sustainability. Comparisons were made between glass-made vessel photobioreactor (PBR) and NPBR in view of biomass and lipid production, as well as the pollutants removal efficiencies from POME.

## 2. Materials and methods

### 2.1 Novel-designed photobioreactor characterization

A flat panel photobioreactor was designed and applied to the study (Figure 1). The photobioreactor was made up of acrylic material which was transparent for the entire unit setup. The dimension of the photobioreactor was *V*_*R*_ = (40 cm length × 3 cm width × 60 cm height) – (0.5 × 40 cm base × 3 cm width × 3 cm height), with 7.02 L of working volume. The reduction shown in *V_R_* calculation indicates the reduction in volume due to the triangular shape-based photobioreactor. The reactor thickness should be as small as possible, so as to promote light penetration. The thickness of 48 mm and 24 mm gave higher yields than in 90 mm [12]. The walls of the photobioreactor were very thin, with only 3 cm. This was designed to ensure sufficient and effective light illumination. The design of photobioreactor involves *A_R_* per *A_G_* ratio to be in the range of 10 or higher. *A_R_* in m^2^ represents the total transparent area part of the reactor to receive light; whereas *A_G_* in m^2^ represents the ground level of the reactor which measures the light energy is collected. The *A_R_* per *A_G_* ratio was 60, therefore representing the great efficiency of the whole unit to receive light per small ground area required. Flat panel photobioreactor provides a high surface per volume ratio (SVR) to capture more solar energy per volume basis. The SVR of photobioreactor is commonly found less than 100 m^2^/m^3^, while for an open pond is less than 4 m^2^/m^3^. Typical SVR ratios are 80 to 100 m^2^/m^3^ for flat plate, bubble column and tubular photobioreactor [12]. SVR of the photobioreactor was 73.37 m^2^/m^3^, which was closed to the SVR of commercial-scale flat-panel photobioreactor. The photobioreactor was continuously illuminated using an external light source (220–240 V fluorescent lamps; Bistar Lighting Co., Ltd). This external light source was mounted on both sides of the photobioreactor. The light intensity used was set at about 8000 lux, measured at the top, middle and bottom part of the photobioreactor. The light intensity on the reactor wall was measured using Lutron Lux meter LX-103. The photobioreactor was operated at a temperature of 25°C, throughout the cultivation cycle. The CO_2_ concentration supplied was with 2.5% mixture with atmospheric air, in compressed gas form. The photobioreactor was installed with a check valve, to ensure the flow of CO_2_ only in one direction therefore preventing back flow. The photobioreactor was also installed with a gas diffuser to promote proper mixing of bubbles into the medium. A gas diffuser also provides small bubbles with overall larger surface areas, thus making cell contact with CO_2_ more efficient. The bubbling using diffuser was supplied by compressed CO_2_, negating any cost attributed to bubbling and pumping. The gas holdup is described by the volume fraction of gas phase within the gas bubbles [13]. The gas holdup was minimal with bubbles diffuser, creating small bubbles which are retained by the baffles within the photobioreactor. The baffles are installed in the photobioreactor, so as to ensure longer retention time of bubbles within the culture medium. The mixing of the biomass is dependent on bubbles movement. This ensures no shear stress is imposed on the biomass in the photobioreactor. Agitation with bubbles is a more gentle technique with regards to cell stress [12]. The triangular shape of the bottom of the photobioreactor serves to ease microalgae cell harvesting by sedimentation. Liquid samples were collected daily for determination of the biomass concentration as well as lipid, the latter of which was collected at set time intervals.

**Figure 1.** Schematic representation (a) and real picture (b) of novel-designed photobioreactor.

### 2.2 Medium compositions, microalgae preculture, determination of biomass concentration, lipid content and pollutant removal efficiencies

The details of analytical methods are summarized in our previous work [14–16]. Microalga species *Chlorella sorokiniana* CY-1 was used in the present study. Sterile BG11 medium was used to preculture the CY-1 for 5 days. The PBR used was 1 L glass-made vessel. The glass vessel PBR was continuously illuminated using an external light source, mounted on both sides of the PBR. 8000 lux light intensity was applied. The PBR was operated at 25°C, supplied with 2.5% and 0.1 vvm CO_2_ aeration. After 5 days of preculture, microalgae cells are concentrated by centrifugation. The inoculum ratios of CY-1: *Pseudomonas* sp. of 1:1 were incorporated for cultivation as described in [16]. The medium applied was 30% [v/v] POME-water culture medium, supplemented with 200 mg L^−1^ of glucose, urea and glycerol. The media were autoclaved prior to its use for cultivation. Daily sampling carried out to determine the dried microalgae biomass concentration. Aliquots of 5 mL culture was sampled and microalgae cells were collected using centrifugation as described in [17]. The sample was then be resuspended in water in crucible and being dried at 105°C to obtain the constant weight. Triplicates of samples were analyzed. For lipid content determination, microalgal cells were harvested and undergone freeze-drying to obtain dried biomass at intervals. Transesterification is the direct conversion reaction of triglycerides into fatty acid methyl esters (FAMEs). The lipid content and compositions were determined as FAMEs after transesterification [18]. The samples were analyzed using GC-FID. The wastewater characteristics chemical oxygen demand (COD), total nitrogen (TN) and total phosphorus (TP) were determined following the American Public Health Association on Standard Methods on the examination of water and wastewater.

## 3. Results and discussion

### 3.1 Comparison between glass-made vessel and novel-designed photobioreactor: biomass concentration and productivity

Biomass concentration and productivity of *Chlorella sorokiniana* CY-1 cultivated in scale-up glass-made vessel of 5 L photobioreactor and novel-designed photobioreactor were compared. As shown in Figure 2(a), the maximal biomass concentrations obtained in NPBR and glass-made vessel PBR were 5.74 g L^−1^ and 2.50 g L^−1^, respectively, on day 20. Besides, the biomass productivities were 408.9 mg L^−1^ d^−1^ and 228.9 mg L^−1^ d^−1^, respectively, for the former and latter (Figure 2(b)). Significant improvement was obtained, indicating the effectiveness of NPBR in biomass production, as compared to 5 L glass-made vessel PBR. The major differences in the design include the thickness of the NPBR which was only 3 cm, as well as a larger transparent surface area which enables shorter light path through the POME medium. On the contrary, 5 L glass-made vessel has a diameter of 18.2 cm, with a height of 33.5 cm. Effective illumination brings higher photosynthetic efficiency [19]. The glass-made vessel PBR was 6 times larger in diameter, compared to the thickness of NPBR. Cultivation using dark color wastewater cause photolimitation, with low light received for cells location the center region [20]. In addition to better light penetration, microbubbles generated with retention using baffles in NPBR provide better CO_2_ supply. As reported by Lam et al. [21], microbubbles have lower rising velocity, and their size gradually decreases as they rise to the surface of the liquid medium, bursting as they reach the surface. On the other hand, macrobubbles rise more rapidly and usually collapse after reaching the surface of the liquid medium. With both the retention and generation of the microbubbles, the latter mostly burst in the culture medium. NPBR ensures effective utilization by microalgae in the culture medium. The CO_2_ utilization is reduced by at least 50% as compared to CO_2_ supply in glass-made vessel PBR in this study. Apart from this, microbubbles also provide higher surface area to volume ratio, enabling effective microalgae cell contact with CO_2_. Membrane photobioreactor, due to the microbubbles concept, is apparently becoming the popular photobioreactor applied to the microalgae industry [21]. The biomass concentration and productivity attained were successfully optimized using the innovative idea of enhancing illumination and CO_2_ supply.

**Figure 2.** Biomass concentration (a) and biomass productivity (b) of *Chlorella sorokiniana* CY-1 cultivated in scale-up PBR and novel PBR.

### 3.2 Comparison between glass-made vessel and novel-designed photobioreactor: lipid content

Microalgae samples were collected at intervals along the cultivation cycle, and undergo *in-situ* transesterification and fatty acids quantification using gas chromatography. Lipid content was found to increase along the cultivation cycle. The lipid yields of CY-1 cultivated in NPBR were found to be higher than that cultivated in glass-made vessel PBR, for every sample taken. Figure 3(a) shows the time course profile of lipid content exhibited by *Chlorella sorokiniana* CY-1 cultivated in glass-made vessel PBR and NPBR. The maximal lipid yields exerted were 14.43% and 4.83%, in NPBR and glass-made vessel PBR on day 20. The most significant lipid accumulation attained was on day 20 in NPBR, whereby the lipid content attained was about three folds more than CY-1 cultivated in glass-made vessel PBR. Conversely, the lipid accumulated in glass-made vessel PBR did not show significant improvement in lipid accumulation along the cultivation cycle. This could be due to its overall slow biomass growth along the cultivation cycle, especially after day 10 (Figure 2(a)). Overall, the results of NPBR shows an increase in effectiveness in both the biomass production as well as the lipid accumulation. High biomass concentration has brought about relatively higher lipid yield. Figure 3(b) indicates the fatty acids composition of *Chlorella sorokiniana* CY-1 cultivated in NPBR on day 20. The highest percentage of C15 (52.67%), followed by C18 (29.66%) and C16 (24.89%) was obtained. The ideal fatty acids are C16 and C18 for biodiesel production, whereas C15 works well for biokerosene. In the present study, the FAME compositions were predominated by C15, with 52.67%. The C16 and C18 were about 30% each. This indicated that the CY-1 could be potentially used for biofuel production at a larger scale including biokerosene production.

**Figure 3.** Lipid content (a) of *Chlorella sorokiniana* CY-1 cultivated in glass-made vessel and novel PBR and FAME compositions (b) of *Chlorella sorokiniana* CY-1 cultivated in novel PBR at day 20.

### 3.3 Comparison between glass-made vessel and novel-designed photobioreactor: pollutants removal efficiencies in POME

The internal composition of the microalgae cell is C:N:P for 106:16:1 following Redfield ratio [22,23]. This ratio is representing the important element required by microalgae for effective growth. Nitrogen is vital for microalgal nucleic acid and protein synthesis, while phosphorus is necessary for ribosomal RNA synthesis [23,24]. These pollutants assimilation would also be representing the pollutants removal from the wastewater. Xiong et al. [25] has recently studied the practical feasibility of using microalgae to remove pharmaceutical contaminants [25]. Modified algae can also be applied for heavy metals removal [26]. Figure 4 shows the pollutants removal efficiencies of *Chlorella sorokiniana* CY-1 cultivated in glass-made vessel PBR and novel PBR. The pollutants were removed very efficiently NPBR, with removal efficiencies of 93.7% of COD, 98.6% of TN and 96.0% of TP. Conversely, in the glass-made vessel PBR, CY-1 also attained high performance too in TN and TP removal, at 96.6% and 98.0%, respectively. However, the COD removal was only 55.1% in glass-made vessel PBR, which was lower than the 93.7% removal efficiency in NPBR. Overall, it could be concluded that the pollutant removal efficiencies achieved by CY-1 cultivated in NPBR were greater than that of the glass-made vessel PBR, for the pollutants of concern. This was due to the overall excellent performance of biomass growth in NPBR, which assimilated lots of pollutants from wastewater. The biomass achieved in NPBR was more than 2 folds yield compared to the glass-made vessel PBR. More organics were assimilated in the former, leading to a high COD removal efficiency. TN and TP also appeared to be more easily assimilated than the carbon source. The present results showed that cultivating CY-1 in NPBR yields an excellent pollutants removal percentage with a high performance of biomass and lipid production.

**Figure 4.** Pollutants removal efficiencies of *Chlorella sorokiniana* CY-1 cultivated in glass-made vessel PBR and novel PBR.

Table 1 summarizes the comparative studies on biomass and lipid yields of *Chlorella* sp. cultivated in POME. The biomass production of CY-1 cultivated in novel-designed PBR achieved excellent results compared to our previous work, which was cultivated at a smaller scale (1 L) using lab flask method, with the same cultivation medium. However, the lipid yield obtained was lower in NPBR. This could be due to the scaling up effort, which has more controlling factors compared to the lower scale study. Moreover, high biomass production did not always bring about a high lipid accumulation as more energy could be used up for cell duplication rather than energy reserve in the lipid accumulation. Yet, the overall biomass and lipid yields obtained in this study showed significantly higher biomass growth and lipid production as compared to the studies found in the literature. It should also be noted that Ponraj and Din [27] have reported a high biomass concentration up to 39.41 g L^−1^ due to the difference in the PBR system, which was using a programmable-controlled reactor tank applied for *Chlorella* sp. cultivation.

**Table 1.** The biomass and lipid yields of microalgae species grown in POME.

No.	Microalgae strain	Culture medium	Cultivation method	Maximal biomass concentration (g L^−1^)	Growth rate (d^−1^)^a^ Biomass productivity (g L^−1^ d^−1^)	Lipid content (%)	Nutrients reduction	References
1	*Chlorella sorokiniana CY-1 + *Pseudomonas* sp. at ratio 1:1*	30% (v/v) POME + 200 mg L^−1^ glucose + 200 mg L^−1^ glycerol + 200 mg L^−1^ urea	Novel-designed PBR	5.74	408.90	14.43	Removal of 93.7% COD, 98.6% TN, 96.0% TP	This study
2	*Chlorella sorokiniana CY-1 + Pseudomonas sp. at ratio 1:1*	30% (v/v) POME + 200 mg L^−1^ glucose + 200 mg L^−1^ glycerol + 200 mg L^−1^ urea	Glass-made vessel PBR	2.50	228.90	4.83	Removal of 55.1% COD, 96.6% TN, 98.0% TP	This study
3	*Chlorella sorokiniana* CY-1 + *Pseudomonas* sp. at ratio 1:1	30% (v/v) POME + 200 mg L^−1^ glucose + 200 mg L^−1^ glycerol + 200 mg L^−1^ urea	Lab scale flask	2.04	185.71	16.04	Removal of 53.7% COD, 55.6% TN, 77.3% TP	[16]
4	*Chlorella vulgaris*	POME + 60 mg L^−1^ urea	Lab scale flask	1.07	76.43	-	Removal of 45.08% COD	[28]
5	*Chlorella* sp.	50% (v/v) POME + 1 g L^−1^ urea	Lab scale flask	-	0.06 ^a^	-	-	[29]
6	*Chlorella pyrenoidosa*	10% (v/v) POME	Programmable controlled reactor tank	39.41	-	-	-	[27]
7	*Chlorella vulgaris*	40% (v/v) POME + D-glucose	Lab scale flask	1.43	1.406 ^a^	9.7	-	[30]
8	*Chlorella vulgaris*	40% (v/v) POME + glycerol	Lab scale flask	0.98	0.328 ^a^	7.3	-	[30]

### 3.4 A mathematical model

To better understand the mechanism behind the growth of the microalgae in this work, the Huisman Model [31] is applied. According to the Huisman Model, the density of microalgae $A\left(t\right)\geq 0$ at time t is described by the ordinary differential equation

(1) $$\frac{dA}{dt}=H\left(A\right)\;:=\frac{\mu_{max}}{z_{max}}\ln\left(\frac{H_{p}+I_{in}}{H_{p}+I_{out}}\right)\frac{A}{kA+k_{bg}}-h_{r}A\;\;\;\;\;\;\;\;\;\;\;\;\;\;\;\;\;\;\;\;\;\;\;\;\;\;\;\;\;\;\;\;\;\;\;\;\;\;\;\;\;\;\;\;\;\;\;\;\;\;-D_{r}A$$

where $I_{in}$ is incoming light, $I_{out}$ is outgoing light, $k_{bg}$ is background turbidity, $z_{max}$ is mixing depth, $h_{r}$ is dilution/outflow, $\mu_{max}$ is maximum specific growth rate, $H_{p}$ is half-saturation of photosynthesis, k is specific light attenuation, $D_{r}$ is specific maintenance (death rate). The first and second term on the left-hand side of (1) corresponds to gain and loss of microalgae, respectively.

Assuming zero turbidity and applying Laplace Transform to (1) gives

(2) $$L\left\{\frac{dA}{dt}\right\}=s\overset{ˉ}{A}\left(s\right)-A\left(0\right)=\frac{\frac{\mu_{max}}{z_{max}}\ln\left(\frac{H_{p}+I_{in}}{H_{p}+I_{out}}\right)-\left(h_{r}+D_{r}\right)k_{bg}}{ks}-\left(h_{r}+D_{r}\right)\overset{ˉ}{A}\left(s\right)$$

Solving (2) gives

(3) $$\overset{ˉ}{A}\left(s\right)=\frac{\frac{\mu_{max}}{z_{max}}\ln\left(\frac{H_{p}+I_{in}}{H_{p}+I_{out}}\right)-\left(h_{r}+D_{r}\right)k_{bg}}{ks\left[s+\left(h_{r}+D_{r}\right)\right]}\;\;\;\;\;\;\;\;\;+\frac{A\left(0\right)}{s+\left(h_{r}+D_{r}\right)}$$

Reverting (3) back to t domain gives

(4) $$A\left(t\right)=\frac{\alpha -\beta k_{bg}}{\beta k}+\left[A\left(0\right)-\frac{\alpha -\beta k_{bg}}{\beta k}\right]e^{-\beta t}$$

where $\alpha =\frac{\mu_{max}}{z_{max}}\ln\left(\frac{H_{p}+I_{in}}{H_{p}+I_{out}}\right)$ and $\beta =h_{r}+D_{r}$. α and β are factors affecting the rate of increase and decrease of microalgae, respectively; α corresponds to an increase in microalgae due to light, and β corresponds to a decrease in microalgae due to dilution/outflow and death. From (4), if

(5) $$\frac{\alpha }{\beta }>\left[A\left(0\right)k+k_{bg}\right]$$

$A\left(t\right)$ decreases with time. Else if

(6) $$\frac{\alpha }{\beta }<\left[A\left(0\right)k+k_{bg}\right],$$

$A\left(t\right)$ increases with time but saturates as t→∞ corresponding to Figure 1(a).

Thus, it can be seen from (6) that the light received by the microalgae must be sufficiently greater than a minimum threshold before the algae can be cultivated. In addition, from (6) it can also be deduced that the initial mass of the microalgae plays a major role in successful algae cultivation, and a large enough initial microalgae mass can ensure the cultivation is sustainable.

## 4. Conclusions

Overall, it can be concluded that the cultivation of *Chlorella sorokiniana* CY-1 in POME using novel-designed PBR has brought enhancement in biomass production, excellent lipid content and productivity, as well as effective POME remediation. The glass-made vessel PBR was unable to provide biomass and lipid yields on a larger scale. Thus, the application of the effective design of photobioreactor is effective for larger-scale cultivation. This application has potentially contributed towards more effective biofuel production and wastewater bioremediation, thereby allowing for environmental sustainability.

## Highlights

- *Chlorella sorokiniana* CY-1 grown in POME using novel and glass vessel PBR.
- Biomass and lipid yields were 2.3–2.9 folds higher in NPBR than in PBR.
- Pollutants removal efficiencies were 93.7% (COD), 98.6% (TN) and 96.0% (TP).
